The article "Clinical Research of Orthopedic Trauma Based on Computer 3D Image Analysis" was retracted in 2022. Reason: concerns about the peer review.

# Clinical Research of Orthopedic Trauma Based on Computer 3D Image Analysis

**DOI:** 10.1155/2021/2728388

**Published:** 2021-12-07

**Authors:** Feng Zhao, Jun Fang, Da Li, Qingnan Hong, Ruijin You, Kun Chen

**Affiliations:** Orthopaedics, Quanzhou Strait Hospital, Quanzhou City, Fujian Province, China 362000

## Abstract

In order to improve the clinical research effect of orthopedic trauma, this paper applies computer 3D image analysis technology to the clinical research of orthopedic trauma and proposes the BOS technology based on FFT phase extraction. The background image in this technique is a “cosine blob” background image. Moreover, this technology uses the FFT phase extraction method to process this background image to extract the image point displacement. The BOS technology based on FFT phase extraction does not need to select a diagnostic window. Finally, this paper combines computer 3D image analysis technology to build an intelligent system. According to the experimental research results, the clinical analysis system of orthopedic trauma based on computer 3D image analysis proposed in this paper can play an important role in the clinical diagnosis and treatment of orthopedic trauma and improve the diagnosis and treatment effect of orthopedic trauma.

## 1. Introduction

There are many types of trauma and orthopedic injuries, and the same injury cases can be treated differently due to different ages, different hospitalization times, and different injury conditions [1]. Therefore, choosing an appropriate time and standard treatment plan will bring a good prognosis for the patient. However, treatment programs that are not in line with the times and are not standardized can cause physical dysfunction from the slightest to the loss of physical function and lifelong disability and even threaten the life of the patient. Due to the particularity of the anatomical structure and physiological function of the iliac and soft tissues, there is a strong professionalism in the rescue and treatment of fractures. Traditional disease diagnosis is to use the doctor's personal theoretical knowledge and practical experience to comprehensively analyze and reason. Therefore, a large number of experts with solid theoretical foundation and rich experience have emerged at home and abroad, and they have their own expertise and characteristics [2]. However, the improvement of the level of young physicians largely depends on theoretical knowledge in books and personal exploration, as well as the richness of the cases encountered and the clinical teaching of medical experts. Therefore, there is a certain degree of one-sidedness and subjectivity in diagnosis. How modern orthopedic doctors, especially the vast number of primary medical workers, can reasonably use such huge expert knowledge and practical experience to deal with the ever-changing injuries and diseases in their busy work, give each case the most reasonable treatment method at the best time to achieve the most ideal treatment effect, effectively reduce the occurrence of clinical misdiagnosis and mistreatment, and avoid medical errors and clinical medical disputes is a problem that needs to be solved at present [3].

The article "Clinical Research of Orthopedic Trauma Based on Computer 3D Image Analysis" was retracted in 2022. Reason: concerns about the peer review.

In recent years, due to the rapid development of computer database technology, image processing technology, and network technology, many achievements have been made in military, petroleum engineering, geological exploration, Kaoji discovery, navigation and aviation, and medical diagnosis and treatment. Clinical medical diagnosis and treatment are an important part of various fields of medicine and health. Its development will bring rapid development to the medical and health industry. Computer-aided technology will bring the accuracy, safety, system, and large capacity of calculations into the medical and health field. With the rapid development in clinical data retrieval and collection, medical data statistics, bed monitoring disease diagnosis and treatment, auxiliary surgical positioning, etc., sophisticated modern clinical orthopedic physicians can quickly and accurately diagnose limb trauma without the presence of trauma orthopedic experts. It is imperative to make a corresponding treatment plan based on the diagnosis. The introduction of computerized artificial intelligence systems into the field of orthopedics makes it possible to solve such problems. We can use computers to organize the professional knowledge and practical experience of human experts into a knowledge base to make it achieve systematization, completeness, and production of expert system software which can not only make full use of these precious sources but also avoid the disappearance of such knowledge due to the aging of experts.

Traumatology and orthopedic expert system is an important branch of artificial intelligence medical application. The theory and methods of artificial intelligence (such as knowledge key storage, reasoning judgment, and output) are mainly applied in the form of expert system. The research and development of expert system and the theory of artificial intelligence have been continuously enriched and developed. The orthopedic trauma expert system facilitates the absorption, preservation, and application of the valuable expertise and clinical experience of modern orthopedic experts, to more effectively exert the potential of clinical orthopedic doctors and overcome the contradictions that clinical orthopedic experts lack. The orthopedic expert system as a kind of computer inherits the fast and accurate characteristics of computers and is more reliable and flexible than human orthopedic experts in some aspects and can be free from the influence of time, region, and human factors. The orthopedic traumatology expert system can synthesize the knowledge and experience of many orthopedic experts, including the knowledge input by experts, books, and self-summary, so as to learn from others' strengths, provide high-quality diagnosis and treatment methods, and comprehensively utilize various orthopedics. The knowledge of experts thereby expands and extends the intelligence of human orthopedic experts.

The article "Clinical Research of Orthopedic Trauma Based on Computer 3D Image Analysis" was retracted in 2022. Reason: concerns about the peer review.

This article combines computer 3D technology to analyze the clinical images of trauma and orthopedics and provides a reference for subsequent clinical research in trauma and orthopedics.

## 2. Related Work

Medical images contain a wealth of information, and doctors are accustomed to use this information to diagnose diseases. However, when these images are used at the surgical site, they are not the best choice. The current images produced by CT, MRI, X-ray, etc. only contain two-dimensional information. Therefore, doctors need to rely on experience to restore this two-dimensional information and the relative positions of surgical instruments at different times from time and space. In traditional surgery, doctors use experience to design surgical plans, record or describe them in a rough way, and then perform operations based on impressions [4]. The quality of this kind of surgical plan depends on the individual doctor's surgical clinical experience and skills, and the concept of the surgical plan maker is not easy to be intuitively understood by others. In addition, the redundancy and distortion of the image information affect the efficiency of the entire system. Many image processing problems in surgical navigation systems include image segmentation, three-dimensional image reconstruction, and registration fusion. Image segmentation is the process of recognizing and reorganizing local regions with similar characteristics and is a key step in image processing. Moreover, image segmentation can use statistical classification, threshold, edge detection, area detection, and other techniques [5]. Through image segmentation, the extraction of various tissues such as bones and soft tissues is completed, and the structure and spatial position of different tissues are obtained, and the information required by the doctor is provided in the most concise and clear way. Through three-dimensional image reconstruction, two-dimensional information can be converted into three-dimensional information, so as to help doctors restore the three-dimensional shape of various tissues. Through the registration and fusion of different modal medical images, the advantages of various diagnostic images can be fully expressed. For example, CT images can clearly display the information of bone tissue, MRI images are more expressive for soft tissues, and fMRI and PET can express information about tissue functional areas. This information can help doctors develop a better surgical route with less loss [6].

The article "Clinical Research of Orthopedic Trauma Based on Computer 3D Image Analysis" was retracted in 2022. Reason: concerns about the peer review.

The goal of the three-dimensional positioning system of surgical navigation is to obtain the three-dimensional coordinates of the patient entity and the surgical instrument in its measurement range in real time, so as to determine the spatial position of the patient and the surgical instrument. The accuracy of spatial positioning is directly related to the accuracy of the surgical navigation system, related to the success or failure of the operation under the navigation system, and is one of the key technologies of the surgical navigation system [7]. The spatial positioning technology of the surgical navigation system has undergone a development process from framed to frameless. The operation of surgical navigation with framed spatial positioning is tedious and time-consuming, and the accuracy is limited. Taking neurosurgery intracranial surgery as an example, it is necessary to drill and nail the bone plate outside the patient's head and add a fixed head frame, which will cause pain to the patient and affect the implementation of surgical operations in a certain area [8].

Frameless space positioning has become the mainstream. According to different principles, frameless spatial positioning technology can be divided into robotic arm positioning method, ultrasonic positioning method, electromagnetic positioning method, and optical positioning method [9]. Robotic space positioning method is a contact measurement method, which was first applied to frameless positioning devices. The spatial positioner is composed of a passive mechanical arm with 6 degrees of freedom, and each joint has an encoder formed by a potentiometer. The position and posture of the end of the passive arm (or connected tool) can be determined by the geometric model of the mechanical arm and the encoder. The output value is calculated in real time [10]. The robot arm positioner has a high spatial positioning accuracy, which can reach within a millimeter, but it is relatively heavy and troublesome to install. In addition, because it needs to contact the patient, there is a problem of disinfection of the equipment. Ultrasonic measurement is a noncontact measurement [11]. Based on the measurement of ultrasonic propagation time, it can detect the position of multiple points or multiple rigid bodies without obstructing the operation area. Temperature, humidity, airflow, and the size of the transmitter are the main factors affecting accuracy. It is generally considered that the ultrasonic positioning method has the lowest accuracy [12]. The electromagnetic locator contains 3 magnetic field generators. Each magnetic field generator coil defines a spatial direction. The detector coil detects the low-frequency magnetic field passing through the air or soft tissue. The relative position relationship of the generators can determine the spatial position of the detector. In target positioning, the electromagnetic positioner is low in cost, and there is no light path blocking between the detector and the generator, which is suitable for positioning requirements when the target point is located in the patient's body, such as the positioning of puncture needles and interventional catheters. However, the ferromagnetic material in the surgical area will interfere with the positioning magnetic field, resulting in a decrease in positioning accuracy [13]. The InstaTrak surgical navigation system of GE in the United States adopts the electromagnetic tracking method. The optical positioning method is currently the most widely used positioning method in navigation systems, and its positioning accuracy is higher (second only to the robotic arm method) [14]. Optical positioning uses a camera to observe the target and then uses the principle of binocular vision to reconstruct the spatial position of the target. According to whether the observed target actively emits light, it can be divided into two types: active and passive. Optical locator is the current hot spot of positioning system research; especially, passive optical locator is the mainstream of spatial positioning method in navigation system [15].

The article "Clinical Research of Orthopedic Trauma Based on Computer 3D Image Analysis" was retracted in 2022. Reason: concerns about the peer review.

## 3. 3D Image Analysis Technology of Traumatology and Orthopedics

The background schlieren technology, like other traditional schlieren technologies, also determines the refractive index change of the flow field by measuring the amount of light deflection and then obtains the density change of the flow field. The relationship between the refractive index and density of a fluid can be expressed by the Lorentz-Lorenz equation:

(1) $$\begin{array}{c} \frac{n^{2}-1}{n^{2}+2}=\frac{4\pi }{3}N\alpha . \end{array}$$

Among them, *n* is the refractive index, *N* is the number of molecules per unit volume, and *α* is the average polarizability. For gases, the Lorenz-Lorenz equation can be simplified to the Gladstonc-Daleequation:

(2) $$\begin{array}{c} n-1=K\rho , \end{array}$$

where *n* is the refractive index, *K* is the Gladstone-Dale constant, and *ρ* is the density. It gives the quantitative relationship satisfaction between the refractive index and density of the gas. Therefore, only by measuring the refractive index of the fluid the density can be obtained. The background schlieren technology obtains fluid density by measuring the refractive index of the fluid.

Figure 1 is a schematic diagram of the principle of the background schlieren technology. On the far left is the background board, which has a specific pattern—background image, and on the far right is a CCD camera for taking pictures. In the middle of them is the flow field to be measured. The dotted line between the background plate and the CCD camera represents the light when there is no flow field, and the solid line represents the light when there is a flow field. *L*_*A*_ is the distance between the CCD camera and the flow field, *L*_*B*_ is the distance between the CCD camera and the background plate, *L*_*D*_ is the distance between the flow field and the background plate, and *ε*_*y*_ is the deflection angle of the light in the figure. The displacement of the light in the *y* direction of the photosensitive surface of the CCD camera is Δ*y*, and the focal length of the CCD camera lens is *f* when there is no flow field and there is a flow field as shown in Figures 1 and 2.

According to the geometric relationship, the image point displacement (in the *y* direction) can be obtained:

(3) $$\begin{array}{c} \Delta y={ML}_{D}\tan\varepsilon_{y}. \end{array}$$

Among them, the magnification factor is

(4) $$\begin{array}{c} M=\frac{L_{i}}{L_{B}}. \end{array}$$

Under normal circumstances, the deflection angle *ε*_*y*_ of the light passing through the flow field is very small, and it can be considered that *ε*_*y*_ ≈ tan*ε*_*y*_. Then, formula (3) can be written as

(5) $$\begin{array}{c} \Delta y=\frac{L_{D}\varepsilon_{y}L_{i}}{L_{B}}. \end{array}$$

The deflection angle of the light passing through the flow field is

(6) $$\begin{array}{c} \varepsilon_{y}=\frac{1}{n_{0}}\int \frac{\partial n}{\partial y}dz. \end{array}$$

Among them, *n*_0_ is the refractive index of the air outside the flow field to be measured, and *n* is the refractive index of the flow field. In order to capture clear images, the CCD camera should focus on the background plate. According to the relationship between the object distance and the distance, you can get

(7) $$\begin{array}{c} \frac{1}{f}=\frac{1}{L_{i}}+\frac{1}{L_{B}}. \end{array}$$

Then, according to equations (5), (6), and (7), the relationship between the displacement of the image point and the refractive index of the flow field can be obtained:

(8) $$\begin{array}{c} \Delta y=\left(\frac{L_{D}}{L_{D}+L_{A}-f}\right)\frac{f}{n_{0}}\int \frac{\partial n}{\partial y}dz. \end{array}$$

In the same way, we get

(9) $$\begin{array}{c} \Delta x=\left(\frac{L_{D}}{L_{D}+L_{A}-f}\right)\frac{f}{n_{0}}\int \frac{\partial n}{\partial x}dz. \end{array}$$

The displacement of the image point and the refractive index of the flow field satisfy the quantitative relationship shown in equation (8). Therefore, we can obtain the image point displacement through experiments and then obtain the refractive index distribution of the flow field to be measured. According to the relationship between the refractive index and density given by the Gladstone-Dell equation, the density distribution of the flow field to be measured can also be obtained.

The article "Clinical Research of Orthopedic Trauma Based on Computer 3D Image Analysis" was retracted in 2022. Reason: concerns about the peer review.

Obtaining the displacement vector of the image from two images is very similar to a hot issue in the field of computer vision for many years. Optical flow algorithm is currently an important method of moving image analysis. We designed a new background image—a multiscale wavelet noise image. The optical flow algorithm is used to process the background image to obtain the image point displacement.

The optical flow algorithm has the following three premise assumptions:

1. The brightness of image pixels in adjacent frames is constant
2. The pixels in the adjacent frames of the image will not produce large motion
3. The pixels of the same subimage within the image move in a similar way

We assume that the brightness of the pixel (*x*, *y*) at time t is *I* (*x*, *y*, *t*), after Δ*t* time; that is, at time *t* + Δ*t*, the brightness of the pixel is *I*(*x* + Δ*x*, *y* + Δ*y*, *t* + Δ*t*). When Δ*t*⟶0, according to assumption (1), we know

(10) $$\begin{array}{c} I\left(x+\Delta x,y+\Delta y,t+\Delta t\right). \end{array}$$

By carrying out the first-order Taylor series expansion of equation (10), we can get

(11) $$\begin{array}{c} I\left(x+\Delta x,y+\Delta y,t+\Delta t\right)=I\left(x,y,t\right)+\frac{\partial I}{\partial x}\frac{\Delta x}{\Delta t}+\frac{\partial I}{\partial y}\frac{\Delta y}{\Delta t}+\frac{\partial I}{\partial t}+\varepsilon . \end{array}$$

Among them, *ε* is a high-order infinitesimal term. According to hypothesis (2), it can be seen that the pixel points in the adjacent frame images move very little. Therefore, the high-order infinitesimal term *ε* can be ignored; then, it can be obtained that

(12) $$\begin{array}{c} \frac{\partial I}{\partial x}\frac{\Delta x}{\Delta t}+\frac{\partial I}{\partial y}\frac{\Delta y}{\Delta t}+\frac{\partial I}{\partial t}=0. \end{array}$$

If we set *u* and *v* to be the velocity component in the horizontal direction and the velocity component in the vertical direction of the pixel, then

(13) $$\begin{array}{c} u=\frac{\Delta x}{\Delta t}, \end{array}$$

(14) $$\begin{array}{c} v=\frac{\Delta y}{\Delta t}. \end{array}$$

By substituting equations (13) and (14) into equation (12), we can get

(15) $$\begin{array}{c} \frac{\partial I}{\partial x}u+\frac{\partial I}{\partial y}v+\frac{\partial I}{\partial t}=0. \end{array}$$

That is,

(16) $$\begin{array}{c} I_{x}u+I_{y}v+I_{t}=0. \end{array}$$

Among them, *I*_*x*_, *I*_*y*_, and *I*_*t*_ represent the partial derivatives of the image gray value in the *x*, *y*, and *t* directions, respectively. Equation (16) is called the basic equation of optical flow field, which is written in vector form:

(17) $$\begin{array}{c} \nabla I\cdot U+I_{i}=0. \end{array}$$

Among them, ∇*I* = (*I*_*x*_, *I*_*y*_) represents the gradient of the gray value of the pixel in the image at (*x*, *y*), and *U* = (*u*, *v*) represents the optical flow at (*x*, *y*).

The article "Clinical Research of Orthopedic Trauma Based on Computer 3D Image Analysis" was retracted in 2022. Reason: concerns about the peer review.

Since the optical flow velocity component of the pixel is two-dimensional, there are two variables *u* and *v*, and there is only one constraint condition of equation (16), so the optical flow cannot be uniquely determined. In order to be able to uniquely determine the optical flow, new constraints must be added. Researchers have proposed several new constraints for this.

The Lucas-Kanade optical flow algorithm adds the local smoothness assumption of optical flow as a new constraint. The local smoothness assumption of optical flow assumes that the optical flow velocity vector of all pixels in a certain size window in the image is the same. The Lucas-Kanade optical flow algorithm assumes that the optical flow field not only satisfies the constraints of the basic equation of the optical flow field (that is, equation (16)) but also satisfies the constraints of the local smoothness of the optical flow and solves these two constraints simultaneously.

The estimation error of optical flow is defined as

(18) $$\begin{array}{c} \underset{\left(x,y\right)\in \Omega }{\sum }W^{2}\left(x\right){\left(I_{x}u+I_{y}v+I_{t}\right)}^{2}. \end{array}$$

Among them, *W*^2^(*x*) is the window weight function, and its function is to make the central area of the neighborhood have a greater impact on the constraint than the outer area. The solution of formula (18) is

(19) $$\begin{array}{c} U={\left(A^{T}W^{2}A\right)}^{-1}A^{T}W^{2}B, \end{array}$$

where *t* time point is *X*_*t*_ ∈ *Ω*. *A* = [∇*I*(*X*_1_), ⋯,∇*I*(*X*_*n*_)]^*T*^, *W* = diag[*W*(*X*_1_), ⋯,*W*(*X*_*n*_)]^*T*^, and*B* = −[*I*(*X*_1_), ⋯,*I*(*X*_*n*_)]^*T*^.

The article "Clinical Research of Orthopedic Trauma Based on Computer 3D Image Analysis" was retracted in 2022. Reason: concerns about the peer review.

The advantage of the Lucas-Kanade optical flow algorithm is that it has strong antinoise ability and robustness, high accuracy of the algorithm, and faster operation speed. The disadvantage is that it calculates a sparse optical flow field. In the edge of the moving target and the homogeneous area of the target itself, if the pixel movement is very small, it is difficult for this optical flow algorithm to capture the change of speed information.

The constraints of the Lucas-Kanade optical flow algorithm are more stringent, and it is not easy to be satisfied. If the speed of the object is fast, the constraint conditions will not be established, and the subsequent assumptions will have a large deviation, resulting in a large error in the final optical flow. The Lucas-Kanade optical flow algorithm is based on the assumption of local smoothness and is a local method. Therefore, the optical flow algorithm cannot obtain optical flow information in a uniform area in the image.

Considering that when the moving speed of the object is large, the calculation result of the Lucas-Kanade optical flow algorithm will have a large error. Therefore, we hope to reduce the movement speed of the pixels in the image. So I thought of a simple method-one-reduce the size of the image. Assuming that the resolution of the original image is 800 × 800 and the speed of the object is, then, when the size of the image is reduced to 400 × 400, the speed of the object becomes [16,16]; when the size of the image is reduced to 200 × 200. The movement speed of the object becomes reduced. We can see that when the size of the original image is reduced many times, the Lucas-Kanade optical flow algorithm becomes usable again.

We assume *I*(*x*) = *I*(*x*, *y*). *J*(*x*) = *J*(*x*, *y*) represents the gray values of two adjacent frames of images *I* and *J*, respectively, and the speed of a certain point in image *I* is *u* = (*u*_*x*_, *u*_*y*_)^*T*^. The velocity of the corresponding point in the image *J* is *v* = *u* + *d*. Among them, *d* = (*d*_*x*_, *d*_*y*_)^*T*^ is the moving speed of the image at that point. *w* is the radius of the neighborhood (*w* generally takes 2 to 7 pixels). The error is

(20) $$\begin{array}{c} E\left(d\right)=E\left(d_{x},d_{y}\right)=\overset{u_{x}+w}{\underset{x-u_{x}-w}{\sum }}\overset{u_{y}+w}{\underset{y-u_{y}-w}{\sum }}{\left(I\left(x,y\right)-J\left(x+d_{x},y+d_{y}\right)\right)}^{2}. \end{array}$$

There is an optical flow e that minimizes *E*(*d*).

We reduce the height and width of the image to half of the original each time, reducing the *L* layer in total. At this time, the 0th layer is the original image. If we assume that the speed of a certain point in the original image is *a*, then the speed of the *n*th layer is

(21) $$\begin{array}{c} u^{n}=\frac{u}{2^{n}}. \end{array}$$

We assume that the optical flow is calculated in the *L*th layer; then, the calculation result of this layer is passed to the upper layer, that is, the *L*-1th layer, as the initial value *g* for the optical flow calculation of this layer. The algorithm repeats this step until the 0th layer, which is the original image. For any layer *L*, equation (20) becomes

(22) $$\begin{array}{c} E^{L}\left(d^{L}\right)=\overset{u_{x}^{L}+w}{\underset{x-u_{x}^{L}-w}{\sum }}\overset{u_{y}^{L}+w}{\underset{y-u_{y}^{L}-w}{\sum }}{\left(I\left(x,y\right)-J\left(x+d_{x}^{L},y+d_{y}^{L}\right)\right)}^{2}. \end{array}$$

The calculation result *d*^*L*^ of each layer is passed to the upper layer as the initial value of optical flow calculation through the following equation:

(23) $$\begin{array}{c} g^{L-1}=2\left(g^{L}+d^{L}\right). \end{array}$$

The initial value of the highest layer is generally 0. Iterating in this way can obtain the optical flow value of the 0th layer:

(24) $$\begin{array}{c} d=g^{0}+d^{0}. \end{array}$$

When *A*(*x*, *y*) = *I*^*L*^(*x*, *y*) and *B*(*x*, *y*) = *J*^*L*^(*x* + *g*_*x*_^*L*^, *y* + *g*_*x*_^*L*^), formula (20) becomes

(25) $$\begin{array}{c} E^{L}\left(d^{L}\right)=\overset{u_{x}+w}{\underset{x-u_{x}-w}{\sum }}\overset{u_{y}+w}{\underset{y-u_{y}-w}{\sum }}{\left(A\left(x,y\right)-B\left(x+g_{x}^{L},y+g_{x}^{L}\right)\right)}^{2}, \end{array}$$

(26) $$\begin{array}{c} \frac{\partial E\left(d^{L}\right)}{\partial d^{L}}=-2\overset{u_{x}+w}{\underset{x-u_{x}-w}{\sum }}\overset{u_{y}+w}{\underset{y-u_{y}-w}{\sum }}\left(A\left(x,y\right)-B\left(x,y\right)-\left[\begin{array}{c} \partial B\;\partial B\\ \partial x\;\partial y \end{array}\right]d^{L}\right)\left[\begin{array}{c} \partial B\;\partial B\\ \partial x\;\partial y \end{array}\right]. \end{array}$$

When

(27) $$\begin{array}{c} \left[\begin{array}{c} I_{x}\\ I_{y} \end{array}\right]={\left[\begin{array}{c} \partial B\;\partial B\\ \partial x\;\partial y \end{array}\right]}^{T},\\ \delta I=A\left(x,y\right)-B\left(x,y\right), \end{array}$$

formula (26) becomes

(28) $$\begin{array}{c} \frac{1}{2}\frac{\partial E\left(d^{L}\right)}{\partial d^{L}}\approx \overset{u_{y}+w}{\underset{y-u_{y}-w}{\sum }}\overset{u_{x}+w}{\underset{x-u_{x}-w}{\sum }}\left(\left[\begin{array}{c} I_{x}^{2}\;I_{x}I_{y}\\ I_{x}I_{y}\;I_{y}^{2} \end{array}\right]\cdot d^{L}-\left[\begin{array}{c} \delta I\cdot I_{x}\\ \delta I\cdot I_{y} \end{array}\right]\right). \end{array}$$

If we mark

(29) $$\begin{array}{c} \overset{u_{y}+w}{\underset{y-u_{y}-w}{\sum }}\overset{u_{x}+w}{\underset{x-u_{x}-w}{\sum }}\left[\begin{array}{c} I_{x}^{2}\;I_{x}I_{y}\\ I_{x}I_{y}\;I_{y}^{2} \end{array}\right] \end{array}$$

as *G*, and

(30) $$\begin{array}{c} \overset{u_{y}+w}{\underset{y-u_{y}-w}{\sum }}\overset{u_{x}+w}{\underset{x-u_{x}-w}{\sum }}\left[\begin{array}{c} \delta I\cdot I_{x}\\ \delta I\cdot I_{y} \end{array}\right] \end{array}$$

as *b*, then

(31) $$\begin{array}{c} \frac{1}{2}\frac{\partial E\left(d^{L}\right)}{\partial d^{L}}\approx G\cdot d^{L}-b. \end{array}$$

When the function *E*(*d*^*L*^) takes the minimum value, the optical flow can be obtained:

(32) $$\begin{array}{c} d^{L}=G^{-1}b. \end{array}$$

The main idea of the pyramid L-K optical flow algorithm is as follows. In the first step, the algorithm first constructs a pyramid, the original image is at the bottom layer, and each layer above is obtained by downsampling after smoothing the layer below. When the image size is reduced by a few layers (generally 3 to 5 layers), the motion speed of the highest layer image is small enough to use the Lucas-Kanade optical flow algorithm for optical flow estimation. The algorithm starts the optical flow estimation from the highest layer, and its optical flow component is used as the initial value of the optical flow estimation of the next layer. The initial value of this layer is added to the light component of this layer to perform projection reconstruction. The algorithm iterates in this way until the optical flow field of the zero-layer image (original image) is solved.

The article "Clinical Research of Orthopedic Trauma Based on Computer 3D Image Analysis" was retracted in 2022. Reason: concerns about the peer review.

## 4. Traumatology and Orthopedics Based on Computer 3D Image Analysis

The nonimaging navigation system is suitable for surgery where the anatomical structure is fully exposed, typically total knee arthroplasty. The system uses nonimaging positioning and tracking technology. During the operation, the three-dimensional geometric image of the simulated specimen is used for navigation, as shown in Figure 3.

Taking total knee replacement as an example, a dynamic reference frame needs to be installed on the patient's femur and tibia to establish a reference coordinate system. Through the spatial position of each reference frame and the marking point, the spatial position of the joint head is determined, and then, the motion force line of the femur is determined. The surgeon uses the probe point to take the typical feature points of the exposed femur and tibia, selects the prosthesis accordingly, and determines the cutting direction and the amount of cutting. During the operation, the space positioning system is used to track the reference ship installed on the surgical instrument to realize navigation. The fully open navigation system does not require preoperative CT scans or X-ray images but only needs to be used by the doctor to pick up the characteristic points of the anatomical structure with a probe during the operation.

The article "Clinical Research of Orthopedic Trauma Based on Computer 3D Image Analysis" was retracted in 2022. Reason: concerns about the peer review.

The CT image-based orthopedic surgery navigation system uses preoperative CT scans to reconstruct three-dimensional images and uses the three-dimensional model of bone tissue as imaging data for doctors to make surgical plans and intraoperative navigation. As shown in Figure 4, a reference frame is installed on the affected bone in the operation to construct a reference coordinate system. The reference frame is tracked by the spatial positioning system, and the position of the surgical machine is displayed in real time on the navigation image.

Figure 5 shows an orthopedic navigation system based on two-dimensional fluoroscopy images. The navigation system obtains fluoroscopy images before surgery. However, unlike CT images, fluoroscopy images are obtained in the operating room. In addition, the position relationship between the positioning reference frame and the C-arm CA must be recorded under the monitoring of the optical positioning system. However, there is no need for a C-arm during surgery.

The orthopedic navigation system based on CT image and laser scanning registration is mainly composed of the following parts: (1) surgical navigation tool: it is used to transmit or reflect light signals to determine the position of the surgical tool; (2) position tracking tool: it is an optical positioning system, and it monitors the position of surgical instruments by receiving photoelectric signals; and (3) laser scanning measuring instrument: it scans the exposed bone tissue surface; spatial registration workstation: it displays virtual images and reflects the position of surgical instruments and the image data of the patient.  Figure 6 shows an orthopedic navigation system based on registration of CT images and laser scans. The marker frame RO is used to unify the spatial positioning system and the three-dimensional laser scanner, and SO and EE are reference frames fixed on the affected bone and surgical instruments.

CT image data is a discrete tomographic sequence image with a certain layer spacing, the pixel resolution is less than 1 mm/pixel, and the layer spacing is greater than 1 mm. Generally, it is between 2 and 4 mm. Extracting the tissue surface from CT sequence images requires a series of processes, as shown in Figure 7. First, the algorithm generates some intermediate faults through interlayer interpolation and obtains volume data with the same resolution in all directions. After that, the algorithm separates the interested organization from the volume data containing various organization information through segmentation. Finally, the interested organization can display and provide various useful surface information through various reconstruction methods.

The article "Clinical Research of Orthopedic Trauma Based on Computer 3D Image Analysis" was retracted in 2022. Reason: concerns about the peer review.

After proposing a clinical analysis system of trauma and orthopedics based on computer 3D image analysis, the system is verified. In this paper, a database is constructed from hospital diagnosis and treatment images, and multiple sets of data in the database are identified by trauma orthopedics through the system of this paper, and the bone injury feature recognition and clinical diagnosis and treatment effects are counted. The results are shown in Table 1.

From the above research and analysis, it can be seen that the clinical analysis system of orthopedic trauma based on computer 3D image analysis proposed in this paper can play an important role in the clinical diagnosis and treatment of orthopedic trauma and improve the diagnosis and treatment of orthopedic trauma.

## 5. Conclusion

With the development of computer software and hardware technology and digital image technology, medical image three-dimensional reconstruction and visualization technology came into being. Compared with two-dimensional images, three-dimensional medical images are more intuitive and accurate. Using the knowledge of computer graphics, each organization can be systematically and perfectly expressed in the three-dimensional reconstruction, and doctors can use it to better locate the lesion in space and understand the spatial relationship of each anatomical structure in detail. This study explores the application value of three-dimensional reconstruction and rapid prototyping technology in clinical orthopedic surgery and formulates the steps and methods of bone data extraction, three-dimensional reconstruction, and rapid prototype. Furthermore, this study applies the technology to clinical practice in orthopedics, improves the diagnosis rate of orthopedic diseases, and develops personalized treatment plans for patients. Through research and analysis, it can be known that the clinical analysis system of orthopedic trauma based on computer 3D image analysis proposed in this paper can play an important role in the clinical diagnosis and treatment of orthopedic trauma and improve the diagnosis and treatment effect of orthopedic trauma.

## Figures and Tables

**Figure 1:** Schematic diagram of the background schlieren technology principle.

**Figure 2:** Schematic diagram of the pyramid L-K optical flow algorithm.

**Figure 3:** Orthopedic navigation system without image.

**Figure 4:** Orthopedic navigation system based on CT images.

The article "Clinical Research of Orthopedic Trauma Based on Computer 3D Image Analysis" was retracted in 2022. Reason: concerns about the peer review.

**Figure 5:** Orthopedic navigation system based on two-dimensional fluoroscopy images.

**Figure 6:** Orthopedic navigation system based on CT image and laser scanning registration.

**Figure 7:** CT data processing flow.

**Table 1:** Experimental results of the clinical analysis system of trauma and orthopedics based on computer 3D image analysis.

Number	Feature recognition	Clinical diagnosis and treatment	Number	Feature recognition	Clinical diagnosis and treatment	Number	Feature recognition	Clinical diagnosis and treatment
1	90.30	92.70	24	92.64	85.56	47	93.61	81.11
2	95.03	84.83	25	91.42	91.73	48	91.00	87.72
3	93.96	88.73	26	93.83	87.26	49	95.82	89.10
4	90.98	85.49	27	94.13	88.42	50	95.42	92.20
5	90.46	84.87	28	92.13	81.57	51	94.69	82.56
6	93.07	86.37	29	92.48	89.23	52	94.18	88.85
7	90.67	90.27	30	94.97	82.10	53	92.46	87.92
8	93.26	81.98	31	95.28	84.61	54	93.03	81.52
9	90.67	83.84	32	95.30	86.80	55	95.47	91.45
10	95.83	84.26	33	93.39	90.10	56	92.47	86.58
11	92.65	86.16	34	96.87	90.13	57	90.41	84.72
12	93.32	90.75	35	92.43	88.53	58	95.14	89.08
13	93.93	86.79	36	96.21	84.17	59	90.34	85.35
14	93.38	81.95	37	93.42	85.37	60	91.75	88.97
15	93.56	82.05	38	92.82	82.03	61	96.09	87.89
16	94.84	88.57	39	94.95	85.00	62	95.14	91.72
17	96.97	81.61	40	91.58	87.56	63	95.36	84.16
18	90.04	91.46	41	91.43	90.60	64	95.33	82.15
19	91.34	82.84	42	90.09	85.42	65	94.03	82.39
20	94.68	81.96	43	93.26	87.38	66	92.48	81.65
21	95.78	85.19	44	93.76	89.67	67	93.08	85.19
22	96.83	82.61	45	95.05	89.56	68	95.28	82.40
23	95.60	82.76	46	90.96	91.48	69	96.73	85.30

## Data Availability

The data used to support the findings of this study are included within the article.

## References

[1] Park C., Sugand K., Nathwani D., Bhattacharya R., Sarraf K. M. (2020). Impact of the COVID-19 pandemic on orthopedic trauma workload in a London level 1 trauma center: the “Golden month”. *Acta Orthopaedica*.

[2] Olczak J., Fahlberg N., Maki A. (2017). Artificial intelligence for analyzing orthopedic trauma radiographs. *Acta Orthopaedica*.

[3] Kim J. W., Lee Y., Seo J. (2018). Clinical experience with three-dimensional printing techniques in orthopedic trauma. *Journal of Orthopaedic Science*.

[4] Hubbard E. W., Riccio A. I. (2018). Pediatric orthopedic trauma: an evidence-based approach. *Orthopedic Clinics*.

[5] Jones J., Southerland W., Catalani B. (2017). The importance of optimizing acute pain in the orthopedic trauma patient. *Orthopedic Clinics*.

[6] Shiels S. M., Tennent D. J., Wenke J. C. (2018). Topical rifampin powder for orthopedic trauma part I: rifampin powder reduces recalcitrant infection in a delayed treatment musculoskeletal trauma model. *Journal of Orthopaedic Research*.

The article "Clinical Research of Orthopedic Trauma Based on Computer 3D Image Analysis" was retracted in 2022. Reason: concerns about the peer review.

[7] Schottel P. C., Warner S. J. (2017). Role of bone marrow aspirate in orthopedic trauma. *The Orthopedic Clinics of North America*.

[8] Locker P. H., Arthur J., Edmiston T., Puri R., Levine B. R. (2018). Management of bone defects in orthopedic trauma. *Bulletin of the Hospital for Joint Disease (2013)*.

[9] Stahl I., Katsman A., Zaidman M., Keshet D., Sigal A., Eidelman M. (2019). Reliability of smartphone-based instant messaging application for diagnosis, classification, and decision-making in pediatric orthopedic trauma. *Pediatric Emergency Care*.

[10] Haupt E., Vincent H. K., Harris A. (2018). Pre-injury depression and anxiety in patients with orthopedic trauma and their treatment. *Injury*.

[11] Capo J. T., Egol K. A. (2017). Information on orthopedic trauma fellowships: online accessibility and content. *The American Journal of Orthopedics*.

[12] Maurer E., Wallmeier V., Reumann M. K. (2020). Risk of malnutrition in orthopedic trauma patients with surgical site infections is associated with increased morbidity and mortality - a 3-year follow-up study. *Injury*.

[13] Ilfeld B. M., Ball S. T., Cohen S. P. (2019). Percutaneous peripheral nerve stimulation to control postoperative pain, decrease opioid use, and accelerate functional recovery following orthopedic trauma. *Military Medicine*.

[14] Cooper D. B., Curtiss G., Armistead-Jehle P. (2018). Neuropsychological performance and subjective symptom reporting in military service members with a history of multiple concussions: comparison with a single concussion, posttraumatic stress disorder, and orthopedic trauma. *Journal of head trauma rehabilitation*.

[15] Lybrand K. E., Althausen P. L. (2018). The role of value-based implants in orthopedic trauma. *Orthopedic Clinics*.

